# Time to First Dressing Change after Peripherally Inserted Central Venous Catheter (PICC) Insertion in Breast Cancer Patients

**DOI:** 10.1155/2022/9380796

**Published:** 2022-10-03

**Authors:** Yinghua Zeng, Wenji Li, Xiaojin Li, Lanlan Ma

**Affiliations:** Department of Breast, Southern Hospital, Southern Medical University, 6th Floor, Digestive Building, No. 1838, Guangzhou Avenue North, Baiyun District, Guangzhou, Guangdong, China

## Abstract

**Background:**

Peripherally inserted central catheter (PICC) is the most commonly used infusion route for chemotherapy in Chinese breast cancer patients because of its convenience, ease of operation, and many maintenance sites.

**Objective:**

The objective of this study is to investigate the effect of the first dressing change time on the healing of puncture site and the economic and psychological impact in patients with breast cancer after PICC insertion.

**Methods:**

From April 2020 to October 2020, 120 patients with PICC intubation after breast cancer surgery were selected as the research objects and divided into test group and the control group with 60 cases in each group according to the random number table method. The time of the first dressing change in the control group was routinely performed within 24 hours after PICC catheter placement, while the first dressing change in test group was performed at 48 hours after catheter placement. The effect of the first dressing change time after PICC catheterization on patients after breast cancer surgery was compared between the two groups.

**Results:**

There were significant differences between the two groups in the degree of pain after the first dressing change, the degree of oozing at the puncture site within 1 week, the duration of oozing, and the frequency of maintenance within 3 weeks, cost, depression, and anxiety (*P* < 0.05).

**Conclusion:**

The first dressing change 48 hours after PICC cauterization in patients after breast cancer surgery reduces significantly puncture site bleeding, reduces the frequency of dressing change, and benefits the physical and mental health of patients.

## 1. Introduction

Chemotherapy is one of the main treatment methods for breast cancer patients, but long-term chemotherapy has certain damage and stimulation to the blood vessels of patients. Peripherally inserted central catheter (PICC) is the most popular breast cancer surgery in China due to its convenience, ease of operation, and many maintenance sites. The most common route of infusion for patients after chemotherapy is PICC [1]. China's “Infusion Therapy Nursing Practice Guidelines and Implementation Rules” proposes that the puncture dressing should be changed for the first time within 24 hours after PICC catheterization [2]. However, in clinical observation, it was found that patients with breast cancer after PICC intubation often experienced different degrees of blood oozing at the puncture site for several consecutive days after 24 hours of dressing change [3]. The patient complained of pain at the puncture port and bleeding from the puncture port during the first dressing change. Frequent dressing changes also increase the patient's economic [4] and psychological stress [5, 6].

Some studies have shown that prolonging the first dressing change time of PICC in patients with hematological tumors can reduce the occurrence of bleeding at the puncture point [7]. However, the current research on the time of the first PICC dressing change has not done in-depth research on the effects of pain, psychology, and other aspects of patients. Breast cancer patients are mostly women, with low tolerance to pain, and their psychological state is easily affected by multiple factors [8], and is prone to depression, anxiety, and other emotions [9–11]. In order to improve the overall comfort of breast cancer patients undergoing chemotherapy after PICC intubation, we changed the time of the first dressing change after PICC intubation to explore its clinical, psychological, and economic effects on patients after PICC intubation.

## 2. Material and Methods

### 2.1. Research Object

Patients with postoperative breast cancer who were to undergo PICC placement from April 2020 to October 2020 in the breast department of a large comprehensive tertiary care hospital in Guangzhou, Guangdong Province, were selected for the study, and PICC placement under ultrasound guidance was performed by the same nurse. Inclusion criteria: (1) Patients with postoperative chemotherapy for breast cancer; (2) Age ≧18 years; (3) The patient agrees and cooperates with PICC; (4) The upper limb on the placement side meets the placement conditions; (5) Has basic cognitive ability and communication skills. Exclusion criteria are as follows: (1) postoperative bilateral breast cancer; (2) history of psychological disorders; (3) advanced postoperative metastasis; and (4) preoperative neoadjuvant therapy has been performed. Finally, 120 patients were obtained for the study. All study subjects were numbered according to the order of tube placement and divided into 60 cases each in the control group and test group in a 1 : 1 ratio.

### 2.2. Methods

#### 2.2.1. Insertion Methods and Management

(1) Piercing nurse qualification: more than 10 years in PICC placement practice. (2) PICC: uniform manufacturer, using the 4Fr catheter made by Bard, USA. (3) Puncture site: postoperative healthy upper limb, placement vessel with your vein as the first choice, followed by the median elbow vein and brachial vein. Avoid the damaged skin vessels, and choose 4~8 cm above the elbow for puncture. (4) The procedure of tube placement: B ultrasound-guided puncture was performed using the Seldinger technique, and hemostasis was achieved with sterile gauze during tube placement. The weight of the blooded gauze was measured with an electronic scale, and the weight difference between it and the same size of dry gauze was calculated and recorded as bleeding volume. The puncture port was compressed with a 10 cm ×10 cm sterile gauze block folded in 8 layers to stop bleeding, plus IV3000 sterile transparent dressing for fixation. (5) Confirmation of catheter position: After successful placement, press the puncture site for 30 min, and go to the radiology department to take an orthopantomogram of the chest to determine the position of the catheter tip. The tip of the catheter was located in the lower 1/3 of the superior vena cava, indicating successful catheter placement. (6) Postoperative maintenance: The first changing medical dressings were performed by a trained and qualified nurse within 24-h catheter placement in the control group, while the first changing medical dressings were performed within 24-h catheter placement in the test group. Patients in both groups should be continuously observed for 3 weeks after the first changing medical dressings. If there was no bleeding from the puncture port, loosening of the patch, or discomfort of the rash at the patch, the dressing was changed once a week. Once bleeding from the puncture port is detected, the dressing should be changed at any time until the bleeding stops.

### 2.3. Observation Indicator

1) Degree of bleeding at the puncture site: (i) No bleeding: no bleeding after placement; mild bleeding: a small amount of bleeding can be seen in the dressing at the puncture site after the patient is active; (ii) moderate bleeding: a small or moderate bleeding can be seen at the puncture site when lying still , but not beyond the catheter wall; (iii) Severe bleeding: massive bleeding at the puncture site can be seen along the PICC catheter wall [12]. 2) Duration of bleeding at the puncture site: (i) Grade 0: a small amount of bleeding was seen 24 hours after the dressing was placed, but no fresh blood was seen; (ii) Grade I: bleeding at the puncture site continued for 2-3 days; (iii) Grade II: bleeding at the puncture site for 4-5 days; (iv) Grade III: bleeding at the puncture site for 6 days or more [13]. Patients were assessed for pain at the puncture site at the time of the first dressing change. (4) Generalized Anxiety Disorder Questionnaire (GAD-7): This scale was developed by American scholars Pulitzer et al. [14] and Chineseized by Qu Shan and Shengli [15] and is a concise and effective anxiety self-assessment tool. The scale contains a total of 7 entries and is used to understand the patient's emotional state in the past 2 weeks. The scale is rated on a 4-point Likert scale, with 0 being “not at all,” 1 being “occasionally for a few days,” 2 being “often,” and 3 being “Every day.” The total score ranges from 0 to 21. The Bernbach's alpha coefficient was 0.898, and the retest reliability was 0.856. Patient Health Questionnaire Depression Scale (PHQ-9): this scale, developed by Williams et al. [16] and tested for reliability in Chinese version by Xu Yong et al. [17], is an important tool used to assess depression and contains a total of 9 items to evaluate the subjects' emotional state in the past 2 weeks. The scale was scored on a 4-point Likert scale, with scores ranging from 0 to 3 representing “not at all” to “every day.” The total score of the scale ranged from 0 to 27. The Cronbach's alpha coefficient was 0.833, and the retest reliability was 0.801.

### 2.4. Statistical Analysis

SPSS 26.0 software was used for data analysis in this study, and the measurement data were expressed as mean standard deviation, and the count data were expressed as frequency and percentage. The *t*-test was used for measurement data between two groups (age, number of punctures, number of transfers, and bleeding volume); chi-square analysis was used for count data between two groups (occupation, marital status, side of placement, vascular, platelet abnormalities, and chemotherapy regimen); Wilton rank sum test was used for grade data between two groups (education, monthly income, and TNM stage); anxiety and depression scores of the same patient before and after PICC placement paired *t*-test were used for changes in anxiety and depression scores before and after PICC placement in the same patient. *P* < 0.05 was considered statistically significant.

## 3. Results

### 3.1. Comparison of General Data between Two Groups

A total of 60 cases in the control group and the test group were included in this study. The age of the control group was (45.329.0) years old, and the age of the test group was (48.489.10) years old; there was no significant difference in education, occupation, monthly income, and marriage between the two groups; 30 (50%) cases of left upper limb cauterization in the test group. There were 30 (50%) cases of right upper extremity cauterization. 29 (48.3%) cases of left upper extremity cauterization, and 31 (51.7%) cases of right upper extremity cauterization in the control group. There were no significant differences in the anterior platelet abnormalities and blood loss during cauterization; there were no significant differences in disease stages and chemotherapy regimens between the two groups (see Table 1).

### 3.2. Comparison of Blood Oozing after PICC Incubation between Two Groups of Patients

The bleeding at the puncture site was assessed and graded daily for 1 week after catheter placement in both groups. Within 1 week after catheter placement, there was a statistically significant difference between the control group and the experimental group in the degree of blood oozing at the puncture point every day (*P* < 0.05). The patients in the test group generally had less bleeding at the puncture site, and the proportion of patients without bleeding after cauterization was higher over time, and the difference was statistically significant (*P* < 0.05) (see Figure 1).

### 3.3. The Duration of Bleeding at the Puncture Site and the Pain Score

In the control group, 21.7% of the patients in the control group were grade II, and 65.0% were in grade III; 28.3% of the patients in the test group were in grade II, and 5.0% were grade III. There was a statistically significant difference between the two groups in the classification of the duration of bleeding at the puncture point (*P* < 0.05). The pain score of the first dressing change in the control group was 3.28 ± 1.08 points, and the score in the test group was 1.56 ± 0.65 points (see Figure 2).

### 3.4. Comparison of Anxiety and Depression Scores between the Two Groups of Patients before and after Incubation

The paired *t*-test was used to compare the changes in the anxiety and depression scores of the two groups of patients before and after intubation. It can be seen that the anxiety and depression levels of the patients were reduced after intubation, and the difference was statistically significant (*P* < 0.05); among them, the two scores of the patients in the experimental group decreased more significantly after intubation, and the difference was statistically significant (*P* < 0.05). In the control group, there was no significant difference in anxiety scores before and after intubation (*P* > 0.05). However, the depression score was slightly increased, and the difference was statistically significant (*P* < 0.05) (see Figure 3).

### 3.5. Comparison of Maintenance Frequency and Maintenance Cost between Two Groups of Patients within 3 Weeks

The maintenance frequency and maintenance cost within 3 weeks were compared between the two groups, and the independent samples *t*-test was used for comparison. The maintenance frequency in the control group was higher than that in the experimental group, and the difference was statistically significant (*P* < 0.05). The maintenance cost in the control group was higher than that in the experimental group within 3 weeks, and the difference was statistically significant (*P* < 0.05) (see Table 2).

## 4. Discussion

### 4.1. Effect on Bleeding from the Puncture Site

Some investigators have shown through a study of patients with PICC placement in liver disease that changing medication at an interval of 3 days after placement can reduce the occurrence of local blood seepage [18]. The results of Chen Min et al. showed that the first change of medication 48 hours after PICC placement in patients with hematologic tumors was effective in reducing the bleeding from the puncture site; the study by Ma Yujun et al. [19] compared the bleeding from the puncture site at different times after the first change of medication after placement and showed that prolonging the first change after placement was beneficial in reducing divisional bleeding. The results of Figure 2 show that the degree of bleeding at 48 hours after drug exchange in postoperative breast cancer patients after placement was generally on the mild side, and the percentage of patients who did not bleed after placement was higher over time, which is consistent with the findings of Chen Min and Ma Yujun et al. The first dressing change 48 h after PICC placement in postoperative breast cancer patients is in accordance with the guideline recommendation of 48-h change of gauze dressing [20], which can promote healing of the puncture site and reduce blood leakage from the puncture opening. The rationale is that (i) the 48-h period is still in the period of bacterial multiplication inhibition, while the prolongation of the closure time is more conducive to the repair of fiber glass and granulation tissue, and (ii) it can avoid premature destruction of the blood clot leading to re-injury of the puncture site, which can affect wound healing.

### 4.2. Effect on Patient Pain

This study shows that the pain score of patients who changed the dressing of the puncture port 24 h after the placement was significantly higher than that of the 48-h group. The frequent stimulation of antiseptic solution during changing medical dressings will also increase the pain of patients [21]. Therefore, extending the time of the first dressing change for patients with PICC placement after breast cancer surgery can provide longer time for the healing of the puncture port, avoid the stimulation of the wound that has not yet healed by the disinfectant solution, and reduce the pain of patients.

### 4.3. Psychological Impact

The diagnosis and treatment of breast cancer have a strong negative impact on patients' psychological health, triggering various negative psychological reactions such as stress, depression, and anxiety [22]. For breast cancer patients who have just undergone surgery [23], they are psychologically vulnerable, both from having a physical disability after surgery [24] and from the fear of about to start chemotherapy [25]. It has been shown that the majority of patients have anxiety after PICC placement [26], and in this study, it was found that the change in anxiety and depression scores in the control group after PICC placement in breast cancer patients generally increased by 2-3 points compared to the test group. The reasons for this may be due to the lack of knowledge about PICC placement and the restriction of limb movement on the side of the placement, which put the patients in a state of tension and anxiety, and the leakage of blood from the puncture port after placement, which further increased the depression and anxiety of the patients. Therefore, the first changing medical dressings 48 hours after PICC placement in postoperative breast cancer patients can reduce patients' depression and anxiety, which is of great significance to improve the physical and mental health of postoperative breast cancer patients. Therefore, it is especially important to take effective measures to alleviate the adverse psychological symptoms of patients after incubation. For example, ①introduce the purpose and precautions of incubation to patients before PICC placement, and at the same time, distribute graphic and easy-to-understand publicity materials to enhance the effect of education. ②Respect the patient, understand the patient's psychological state patiently before placement, and give support and encouragement. ③During incubation, pay attention to the patient's feelings, and relieve the patient's tension by chatting with the patient or playing relaxing music. ④Continue to follow up the patient after the placement of the tube, find out the complications, and deal with them in time to relieve their discomfort that may occur during the period with the tube. ⑤Social support: Care for the patient, the patient is given the necessary life care by the family during the period with the tube. Teach patients and their families how to care for them at home during PICC placement, encourage them to participate in the management of PICC catheters, and help patients gain confidence.

### 4.4. Economic Impact

The puncture site should be kept dry and free of blood and fluid after PICC placement. Patients in the control group were changed 24 hours after catheter placement, which led to repeated bleeding at the puncture site after the change because the puncture site had not yet healed and was stimulated by the disinfectant solution during the change. To avoid puncture site infection, the puncture site dressing had to be changed again, so the frequency of maintenance and maintenance costs was higher in the control group patients than in test group. PICC placement operators should standardize the placement process and provide comprehensive and effective health education to patients. Patients and their families should be instructed to continuously observe the puncture site to avoid adverse reactions after placement and to reduce the number and cost of additional hospital admissions for maintenance.

Shortcomings of this study: Pain and bleeding after PICC catheter placement may be related to a variety of factors. This study focused on the effect of the time of the first changing medical dressings after PICC catheter placement and failed to take into account the weight and coagulation of the enrolled patients, and this study was conducted in only one hospital with a small sample size; therefore, it needs to be tested continuously in clinical practice.

PICC catheters provide a safe and effective route to chemotherapy for oncology patients in breast units, but PICC placement requires blade dilation at the puncture port, which inevitably increases injury, and bleeding from the puncture port often occurs after placement [27], and extending the time to the first PICC changing medical dressings is important for postoperative breast cancer patients [28]. The results of this study show that the first changing medical dressings 48 hours after PICC placement in postoperative breast cancer patients can reduce the degree and duration of blood oozing from the puncture port [29].

In conclusion, the first dressing change 48 hours after PICC catheter placement in postoperative breast cancer patients can reduce bleeding at the puncture site, relieve pain, and relieve the patients' depression and anxiety. At the same time, it can also reduce the frequency of dressing changes, reduce the economic burden of patients, and improve the quality of life of patients.

## Figures and Tables

**Figure 1:** Comparison of the degree of bleeding at the puncture port within 1 week after catheter placement between the two groups. In our study, SPSS26.00 statistical software was used for statistical analysis and comparison of the degree of bleeding at the puncture port within 1 week after catheter placement between the two groups. Measurement data expressed as mean ± standard deviation using repeated measures analysis of variance showed that the bleeding at the puncture site was assessed and graded daily for 1 week after catheter placement in both groups. Within 1 week after catheter placement, there was a statistically significant difference between the control group and the experimental group in the degree of blood oozing at the puncture point every day (^∗^*P* < 0.05). The patients in the test group generally had less bleeding at the puncture site, and the proportion of patients without bleeding after cauterization was higher over time, and the difference was statistically significant (^∗^*P* < 0.05).

**Figure 2:** Puncture site oozing duration and pain score. In our study, SPSS26.00 statistical software was used for statistical analysis and puncture site oozing duration and pain score. Measurement data expressed as mean ± standard deviation using repeated measures analysis of variance showed that 21.7% of the patients in the control group were grade II, and 65.0% were grade III; 28.3% of the patients in the test group were grade II, and 5.0% were grade III. There was a statistically significant difference between the two groups in the classification of the duration of bleeding at the puncture point (^∗∗^*P* < 0.05). The pain score of the first dressing change in the control group was 3.28 ± 1.08 points, and the score in the test group was 1.56 ± 0.65 points. Academic differences (^∗∗^*P* < 0.05).

**Figure 3:** Comparison of anxiety and depression scores between the two groups of patients before and after incubation. In our study, SPSS26.00 statistical software was used for statistical analysis and comparison of anxiety and depression scores between the two groups of patients before and after incubation. Measurement data expressed as mean ± standard deviation using repeated measures analysis of variance showed that the changes in anxiety and depression scores of the two groups of patients before and after incubation were compared using paired *t-*test, as shown. The paired *t*-test was used to compare the changes in the anxiety and depression scores of the two groups of patients before and after intubation. It can be seen that the anxiety and depression levels of the patients were reduced after intubation, and the difference was statistically significant. Significant (#*P* < 0.05); among them, the two scores of the patients in the experimental group decreased more significantly after intubation, and the difference was statistically significant (#*P* < 0.05). In the control group, there was no significant difference in anxiety scores before and after intubation (##*P* > 0.05). However, the depression score was slightly increased, and the difference was statistically significant (#*P* < 0.05).

**Table 1:** Table of general patient information [−*x* ± *s*, *n*(%)].

Variables	Control group (*n* = 60)	Test group (*n* = 60)	*P*
Age (years)	45.32 ± 9.07	48.48 ± 9.10	0.059
Education level			
Illiterate	1 (1.7)	2 (3.3)	0.983
Elementary school	14 (23.3)	12 (20.0)	
Junior high school	23 (38.3)	21 (35.0)	
High school/junior college	9 (15.0)	17 (28.3)	
College and above	13 (21.7)	8 (13.3)	
Profession			
Unemployed	18 (30.0)	17 (28.3)	0.240
Self-employed	9 (15.0)	5 (8.3)	
Business unit	7 (11.7)	3 (5.0)	
Staff	20 (33.3)	26 (43.3)	
Retire	6 (10.0)	9 (15.0)	
Monthly income			
<2,000	20 (33.3)	17 (28.3)	0.165
2,000-4,000	28 (46.7)	21 (35.0)	
4,000-8,000	5 (8.3)	18 (30.0)	
>8,000	6 (10.0)	4 (6.7)	
Marriage			
Married	52 (86.7)	57 (95.0)	0.128
Unmarried	6 (10.0)	1 (1.7)	
Widowed/divorced	2 (3.3)	2 (3.3)	
Placement side			
Left	29 (48.3)	30 (50.0)	0.856
Right	31 (51.7)	30 (50.0)	
Blood vessel			
Expensive	56 (93.3)	54 (90.0)	0.511
Brachial vein	4 (6.7)	6 (10.0)	
Number of punctures	1.18 (0.54)	1.13 (0.39)	0.560
Tube times	1.26 (0.70)	1.08 (0.38)	0.093
Bleeding volume (g)	0.76 (0.40)	0.81 (0.30)	0.408
Chemotherapy			
TE	5 (8.3)	2 (3.3)	0.345
TC	1 (1.7)	1 (1.7)	
EC-T	53 (88.3)	56 (93.3)	
Other	1 (1.7)	1 (1.7)	
TNM staging			
0	0 (0.0)	3 (5.0)	0.631
1	4 (6.7)	1 (1.7)	
2	39 (65.0)	36 (60.0)	
3	17 (28.3)	20 (33.3)	

Note: TE is anthracycline combined with taxman; TC is organophosphate combined with taxman; EC-T is anthracycline combined with organophosphate followed by taxman; others are anthracycline combined with taxman followed by platinum.

**Table 2:** Comparison of maintenance frequency and maintenance cost of two groups of patients within 3 weeks.

Variable	Control group (*n* = 60)	Test group (*n* = 60)	*P*
Maintenance frequency	4.80 (1.30)	3.57 (0.85)	<0.001
Maintenance cost (yuan)	443.05 (138.23)	349.25 (86.38)	<0.001

## Data Availability

All data used to support the findings of this study are included in the article.
